# Baicalin Inhibits Inflammation in Rats with Chronic Obstructive Pulmonary Disease by the TLR2/MYD88/NF-*κ*Bp65 Signaling Pathway

**DOI:** 10.1155/2022/7273387

**Published:** 2022-07-22

**Authors:** Jiangang Ju, Zheming Li, Qiang Shi

**Affiliations:** ^1^Department of Respiratory, First People's Hospital of Linping District, Hangzhou 311100, China; ^2^College of Pharmacy, Hangzhou Medical College, Hangzhou 310053, China; ^3^Department of Thoracic Surgery, Hua Mei Hospital, University of Chinese Academy of Science, Ningbo 315010, China

## Abstract

**Objective:**

Chronic obstructive pulmonary disease (COPD) is a chronic inflammatory disease with a relatively high morbidity and death rate. This study aimed to investigate the inhibitory effect of baicalin (BA) on inflammation in COPD rats and its possible mechanism.

**Methods:**

The experimental COPD of SD rats were induced by LPS, smoking, and cold stimulation, and they were randomly divided into the control group, COPD group, COPD + LB group, COPD + MB group, and COPD + HB group. The test of pulmonary function and the HE staining were carried out in COPD rats. The levels of TNF-*α*, IL-1*β*, IL-6, IL-10, and IL-8, as well as GSH, SOD, and MDA in serum, were detected by ELISA. The levels of TLR2, MYD88, TNF-*α,* and IL-1*β* mRNA in BALF were detected by qPCR. The expression of TLR2/MYD88/NF-*κ*Bp65 pathway-related proteins was also detected by the Western blot and immunohistochemistry assays.

**Results:**

Compared to the COPD model group, BA treatment significantly improved the pulmonary function and pathologic changes, reduced the levels of TNF-*α*, IL-1*β*, IL-6, IL-10, IL-8, and MDA, and increased the levels of IL-10, SOD, and GSH in COPD rats. In addition, BA could also decrease the protein levels of MYD88, p–NF–*κ*Bp65/NF-*κ*Bp65, TLR2, and TLR4 but increase the protein level of p-I*κ*Ba/I*κ*B in lung tissue of COPD rats.

**Conclusion:**

BA ameliorated inflammatory response and oxidative stress in COPD rats by regulating the TLR2/MYD88/NF-*κ*Bp65 signaling pathway.

## 1. Introduction

Chronic obstructive pulmonary disease (COPD) is a type of chronic bronchitis and/or emphysema characterized by airflow obstruction which could develop into unusual chronic conditions such as pulmonic heart disease and respiratory failure [1]. The incidence of COPD in China is 8.6%, and its prevalence and mortality are increasing year by year [2]. The development of COPD is associated with abnormal pneumonia to harmful gases and harmful particles such as cigarettes and smoking [3]. The main clinical symptoms of COPD are cough, wheezing, and shortness of breath. COPD is mainly a chronic onset, long course of the disease, and later complications such as chronic pulmonary heart disease, respiratory failure, and gastric ulcer, which impact the patient's quality of daily life to a certain extent [4]. Currently, the use of antibiotics and some hormonal drugs only temporarily relieve symptoms [5].

Repeated chronic inflammation of the airway and the resulting airway remodeling is the key pathological factors for the progression of COPD [6]. The study has found that the TLR signaling pathway plays a crucial part in the inflammatory response [7]. TLRs are relevant to innate immune responses in the body. TLR2 and TLR4 are important members of the TLRs family and play a significant part in inflammation [8]. As an important molecule in the TLR signaling pathway, MYD88 participates in the occurrence and development of inflammation by transmitting upstream signaling [9]. The signal transduction of TLR2 and TLR4 can be combined with MYD88 through the corresponding ligands to activate downstream transcription factors such as NF-*κ*B, which initiate the expression of inflammatory mediators [10]. MYD88 and NF-*κ*B are downstream inflammation signal molecules of TLR2, and cigarette smoke-induced TLR2/MYD88/NF-*κ*B signaling in COPD mice is activated [11].

Baicalin (BA) is a flavonoid derived from *Scutellaria baicalensis Georgi* and has antibacterial, anti-inflammatory, antioxidant, anticancer, and other functions [12]. BA can relieve lung injury and also play an important role in clinical medicine [13]. Li et al. [14] found that BA could inhibit inflammation and reduce inflammatory factors, thereby achieving the effect of inhibiting the inflammatory response. It has been shown that BA could reduce the lipopolysaccharide (LPS)-induced periodontitis in rats by curbing the TLR/MYD88/NF-*κ*B signaling pathway [15]. However, the role of BA in COPD and whether it is related to the TLR2/MYD88/NF-*κ*B signaling pathway remains unclear.

Therefore, this study aimed to explore the effect of BA on inflammation in COPD rats and to explore the possible mechanism of its anti-inflammation effect, which is important for finding new treatments for COPD.

## 2. Materials and Methods

### 2.1. Animals and Groups

Male SD rats were obtained from Shanghai Jihui Laboratory Animal Care Co., Ltd. SCXK (Hu) 2017–0012; Shanghai, China, weighed 230–250 g, 6–8 weeks old, and reared in an environment with a temperature of 23–25°C and a humidity of 55–70%. All SD rats were fed a standard diet and allowed free access to water. After 1 week of adaptive feeding, SD rats were randomly divided into 5 groups (*n* = 6): control group, COPD group, COPD + LB (low dosage of BA) group, COPD + MB (middle dosage of BA) group, and COPD + HB (high dosage of BA) group.

### 2.2. COPD Rat Model Establishment and Treatment

A COPD model was established by the combined application of cigarette smoke, LPS, and cold stimulation [16]. Briefly, the rats in the COPD group were treated with LPS (On days 1 and 14, the anesthetized rats received a trachea injection of 200 *µ*g LPS, dissolved in normal saline), smoked (from the 2nd day to the 28th day, except for the 14th day, smoking with cigarette twice a day.), and maintained at −20°C for 5 min/day (from day 22 to day 29). The rats in the COPD group and the control group were given normal saline and a diet. In addition, the control group did not intervene under the same conditions. The COPD + LB group, COPD + MB group, and COPD + HB group were injected with LPS, smoked, stored at −20°C, and then given BA (dissolved in normal saline) 40 mg/kg/d, 80 mg/kg/d, and 160 mg/kg/d every day from the 8th day for 3 weeks [17]. Finally, the rats were sacrificed, and BALF, serum, and lung tissue were collected for subsequent experiments.

### 2.3. Evaluation of Lung Function

After the last administration, the pulmonary function of the rat was tested with an animal lung function testing machine (Emka France, GYD-003). The mice were placed in a sealed box, connected to a sensor and computer, and acclimated to it for 5 min. Subsequently, lung function was assessed, including functional residual capacity (FRC), forced vital capacity (FVC), peak expiratory flow (PEF), minute volume (MV), forced expiratory volume within 100 ms, and peak inspiratory flow (PIF), and the ratio of FEV100/FVC were calculated.

### 2.4. ELISA

On the 33rd day, the rat's blood was obtained and centrifugated and serum was collected. The levels of TNF-*α*, IL-1*β*, IL-6, IL-10, IL-8, and GSH, SOD, and MDA in serum were detected by ELISA kits.

### 2.5. HE Staining

The right lung of the rat was clamped with hemostatic forceps, then the right lung was removed, fixed with 4% paraformaldehyde, embedded in paraffin, and cut into 4 *μ*m sections. Five specimen sections were taken from each group for HE staining, and pathological changes were observed. Histopathological changes were observed and photographed after HE staining. According to the results of HE staining, it was divided into 5 grades, 0–4 points, respectively [18]. The infiltration of inflammatory cells in rat lung tissues was mainly evaluated, and the higher the evaluation score, the more infiltration of inflammatory cells.

### 2.6. qPCR

Trizol reagent (Vitality, B511311) was used to extract total RNA from rat BALF. Reverse transcription was then performed to synthesize cDNA. Then, the cDNA was analyzed (SYBRPremixExTaq (Takara)). The relative mRNA levels of TLR2, MYD88, and TNF-*α* in BALF were determined with qRT-PCR and calculated according to the 2^−ΔΔCt^ method. The internal reference was GAPDH. The primer sequences used are shown in Table 1.

### 2.7. Immunohistochemistry

The levels of NF-*κ*B, TLR2, and MYD88 in lung tissues were tested using immunohistochemistry. Paraffin-embedded rat lung tissue sections were deparaffinized to water, antigen retrieval was performed in citrate buffer of pH 6.0, and microwave treatment was performed for 20 min. The sections were placed in a 3% H_2_O_2_ solution, incubated at room temperature in the dark for 25 min, and serum-blocked for 30 min. The blocking solution was gently shaken off, and the primary antibodies MyD88 antibody (AF5195, 1 : 125, Affinity), NF-kBp65 antibody (AF5006, 1 : 125, Affinity), and TLR2 antibody (DF7002, 1 : 125, Affinity) were added dropwise to the section and incubated overnight at 4°C. The sections were placed in PBS and shaken 3 times with bleach. After the sections were dried, the secondary antibody (HRP) (S0010, 1 : 200, Affinity) was added dropwise and incubated for 50 min. Then, the slides were washed, and then DAB chromogenic solution was added dropwise to develop color. Finally, hematoxylin was used to stain the slides for 3 min. The slides were rinsed with running water, and then dehydrated and mounted.

### 2.8. Western Blot

The protein expression levels of MyD88, NF-*κ*Bp65, p–NF–*κ*Bp65, I*κ*Ba, p-I*κ*Ba, TLR2, TLR4, and *β*-actin in the rat lung tissue were measured by Western blot. First, the total protein of rat lung tissues was collected, and the total protein concentration was detected by a BCA protein kit (Solarbio, pc0020). The PVDF membrane was blocked by a blocking solution of 5% skimmed milk powder, and the membrane was placed in the incubator box containing the dilution of the primary antibody Anti-MyD88 antibody (AF5195, 1 : 1000, Affinity), Anti-NF-*κ*Bp65 antibody (AF5006, 1 : 1000, Affinity), Anti-p–NF–*κ*Bp65 antibody (AF2006, 1 : 1000, Affinity), Anti-I*κ*Ba antibody (AF5002, 1 : 1000, Affinity), Anti-p-I*κ*Ba antibody (AF2002, 1 : 1000, Affinity), Anti-TLR2 antibody (DF7002, 1 : 1000, Affinity), Anti-TLR4 antibody (AF7017, 1 : 1000, Affinity), Anti-*β*-actin antibody (AF7018, 1 : 10000, Affinity) and incubated it overnight with shaking at 4°C. The next day, the primary antibody was aspirated and washed by TBST 3 times. Next, the membrane was rinsed and horseradish peroxidase-conjugated antibody (HRP) (S0001, 1 : 70000, Affinity) was incubated. Protein bands were detected using an ECL. The secondary antibody (HRP) (S0001, 1 : 3000–1:10000, Affinity) was diluted with a 5% skimmed milk blocking solution and reacted for 1–2 h. The secondary antibody reaction was completed. The bands were visualized by the ECL chemiluminescence instrument development method and chemi capture software. Quantitative analyses were performed using Image J software.

### 2.9. Statistical Analysis

SPSS 19.0 statistical software was used for data analysis. One-way ANOVA analysis of variance was used to measure data across multiple groups, and the SNK test was used for comparison between groups. The Kruskal–Wallis H test was used for variance. All data were expressed as mean ± standard deviation. *P* < 0.05 suggested that the difference was statistically significant.

## 3. Results

### 3.1. BA Improved the Lung Function in COPD Rats

The results of pulmonary function indicators detected by the respiratory function tester are shown in Figure 1. Compared with the control group, the FRC of the COPD group was significantly increased (*P* < 0.01), but the FVC, FEV100, PEF, PIF, and FEV100/FVC were significantly decreased (*P* < 0.01). On this basis, different concentrations of BA were given, and it was found that BA could reverse the results of the above pulmonary function indicators of COPD rats in a concentration-dependent manner.

### 3.2. BA Decreased the Levels of TNF-*α*, IL-1*β*, IL-6, and IL-8 but Increased the Level of IL-10 in the Serum of COPD Rats

The changes of inflammatory factors in the serum of rats were detected by ELISA. The results shown in Figure 2 showed that the levels of TNF-*α*, IL-1*β*, IL-6, and IL-8 in the COPD group were higher than those in the control group (*P* < 0.01), but the content of anti-inflammatory factor IL-10 was lower than the control group (*P* < 0.01), indicating that there was an inflammatory response in the COPD group. After administering BA, the levels of TNF-*α*, IL-1*β*, IL-6, and IL-8 in the serum of rats in each group were significantly reduced (*P* < 0.05 or *P* < 0.01), and the content of IL-10 was significantly increased (*P* < 0.01). It suggested that BA treatment could reduce the inflammatory response in COPD rats.

### 3.3. BA Improved the Levels of Antioxidant Factors in Serum of COPD Rats

The results of serum antioxidant factors detected by ELISA were shown in Figure 3, which showed that the levels of GSH and SOD in the COPD group were significantly lower than those in the control group (*P* < 0.01), and the content of MDA was significantly higher than that in the control group (*P* < 0.01). After giving different concentrations of BA, it was found that the levels of GSH and SOD were higher than those in the COPD group (*P* < 0.05 or *P* < 0.01), and the levels of MDA were lower than those in the COPD group (*P* < 0.01).

### 3.4. BA Improved the Pathological Changes of Lung Tissue in COPD Rats

The pathological changes in rat lung tissues were observed by HE staining. It can be seen from Figure 4 that the bronchial structure of the control group was normal, the airway epithelial cells were clear and intact, and there was no hyperplasia or hypertrophy. However, there were a large number of inflammatory in the lung tube wall and alveolar interstitium in the COPD group. The bronchial mucosal folds increased, the tube wall became thickened and destroyed, the lumen decreased, and the airway epithelial cells proliferated disorderly. When given different concentrations of BA, the lung tissue morphology and structure of the COPD + LB group did not change significantly, and the COPD + MB group and COPD + HB group had complete lung tissue structure, clear alveolar cavity, no inflammatory cell infiltration, and no edema or widening of the alveolar space. In addition, different concentrations of BA significantly reduced the HE semiquantitative score (*P* < 0.01).

### 3.5. BA Reduced the Levels of TLR2, MYD88, TNF-α, IL-1β mRNA in BALF Cells of COPD Rats

The levels of TLR2, MyD88, TNF-*α,* and IL-1*β* mRNA in BALF cells were detected by qPCR. The results in Figure 5 show that the levels of TLR2, MyD88, TNF-*α,* and IL-1*β* in the BALF cells of the COPD group were higher than those of the control group (*P* < 0.01). After administering BA, the levels of TLR2, MyD88, TNF-*α*, and IL-1*β* mRNA in the BALF cells of the COPD + LB group were not significantly different from those of the COPD group. However, the levels of TLR2, MyD88, TNF-*α*, and IL-1*β* mRNA in the BALF cells in the COPD + MB group and COPD + HB group were significantly lower than those in the COPD group (*P* < 0.01).

### 3.6. BA Reduced the Expression of NF-κB, TLR2 and MYD88 in Lung Tissue of COPD Rats

To further explore the effects of BA on COPD rats, the expressions of NF-*κ*B, TLR2, and MyD88 in rat lung tissues were detected by immunohistochemistry. The results in Figure 6 showed that the expressions of NF-*κ*B, TLR2, and MYD88 in the COPD group were significantly higher than those in the control group (*P* < 0.01). After administering BA, the expressions of NF-*κ*B, TLR2, and MYD88 in the COPD + MB group and COPD + HB group were significantly lower than those in the COPD group (*P* < 0.05 or *P* < 0.01).

### 3.7. BA Decreased the Protein Levels of MYD88, p–NF–*κ*Bp65/NF-*κ*Bp65, TLR2, and TLR4 but Increased the Protein Level of p-I*κ*Ba/I*κ*B in Lung Tissue of COPD Rats

The expressions of MYD88, p–NF–*κ*Bp65/NF-*κ*Bp65, p-I*κ*Ba/I*κ*Ba, TLR2, and TLR4 protein in rat lung tissue were detected by Western blot. The result in Figure 7 showed that the expressions of MYD88, p–NF–*κ*Bp65/NF-*κ*Bp65, TLR4, and TLR2 in the COPD group were significantly higher than those of the control group (*P* < 0.01), and the expression of p-I*κ*Ba/I*κ*Ba was remarkably lower than that of the control group (*P* < 0.01). After administering BA, the expressions of MyD88, p–NF–*κ*Bp65/NF-*κ*Bp65, p-I*κ*Ba/I*κ*Ba, TLR2, and TLR4 protein in the lung tissues of the COPD + LB group were not significantly different from the COPD group. However, the expressions of MYD88, p–NF–*κ*Bp65/NF-*κ*Bp65, TLR4, and TLR2 in the lung tissues of the COPD + MB group and COPD + HB group were lower than those of the COPD group (*P* < 0.05 or *P* < 0.01), but the expression of p-I*κ*Ba/I*κ*Ba was remarkably higher than that of the COPD group (*P* < 0.05 or *P* < 0.01).

## 4. Discussion

COPD is a chronical respiratory disease characterized by airway obstruction and pneumonia [19]. The main features of COPD are chronical bronchitis, cough, dyspnea, and small airway obstruction [20]. BA has anti-inflammatory and antioxidant effects [21]. It has been found that BA has a certain alleviating effect on pulmonary fibrosis [22]. Our research found that BA had a significant therapeutic effect on COPD, which may be achieved through the regulation of the TLR2/MYD88/NF-*κ*Bp65 signaling pathway.

In the study, based on predecessors [17], a COPD model was established by giving cigarette smoke, LPS, and −20°C cold stimulation. Pulmonary function testing and lung tissue pathological changes are the criteria for diagnosing COPD [23]. We found that the values of FVC, FEV100, PEF, PIF, and FEV100/FVC in COPD rats decreased, but the FRC value increased, which was consistent with the characteristics of COPD and chronical obstructive pulmonary emphysema [24]. In this study, the HE staining method was used to observe the pathological changes in the lung tissues of rats, and it was found that the lung tissues of the COPD rats had a large number of inflammatory cell infiltrations and the semiquantitative scores were relatively high. This is consistent with the results of the COPD animal model established by the predecessors [25, 26]. In addition, it has been found that BA could effectively restore lung function and lung tissue pathological damage in COPD rats. This is consistent with previous research results that BA could improve airway inflammation in COPD rats [19, 27].

COPD rats are prone to some inflammatory characteristics and oxidative stress [19]. In this study, it was found that the levels of TNF-*α*, IL-1*β*, IL-6, IL-8, and MDA in serum in the COPD rats were remarkably increased, but the levels of IL-10, SOD, and GSH were significantly decreased. BA has anti-inflammatory and antioxidant effects [28]. It is reported that BA could improve airway inflammation in rats induced by cigarettes [27]. In addition, BA reduced the levels of the pro-inflammatory factors in acute lung injury [29, 30], which is consistent with the expression trend in our study. After treatment with BA, it could significantly reduce the levels of inflammation and oxidative factors in the serum of COPD rats, and inhibit the inflammatory response and oxidative stress response in rats, which is similar to the results of Wang et al. [17].

The TLR2/MYD88/NF-*κ*B signaling pathway is currently a more recognized pathway to regulate inflammatory cells [31]. A previous study has shown that the TLR2/4 mediated NF-*κ*B pathway could improve lung inflammation in COPD model rats [32]. Li et al. found that the TLR2/MYD88/NF-*κ*B signaling pathway reduced pulmonary fibrosis [33]. In addition, Bai et al. found that BA may promote collagen-induced arthritis by inhibiting the TLR2/MYD88/NF-*κ*B signaling pathway [34]. In our study, when giving BA treatment, it could reduce the levels of TLR2, MYD88, TNF-*α,* and IL-1*β* mRNA, thereby reduce the expressions of MYD88, p–NF–*κ*Bp65/NF-*κ*Bp65, TLR4, and TLR2, indicating that BA could downregulate the TLR2/MYD88/NF-*κ*Bp65 signaling pathway, which is similar to the BA inhibiting TLR2/MYD88/NF-*κ*B signaling pathway to reduce inflammation in fever rats [15, 35].

This study demonstrated that BA inhibited the inflammatory response in COPD rats by regulating the TLR2/MYD88/NF-*κ*Bp65 signaling pathway and improved lung pathological changes and lung function. However, this study also has certain limitations. More clinical studies should be conducted for revealing its mechanism of action and for providing a solid basis for new drug development. In addition, due to the relatively large number of groups, no positive control experiment was designed. We will design a positive control in the follow-up experiments to make the study more rigorous.

## 5. Conclusion

In summary, the COPD model was established through the combined application of cigarette smoke, LPS, and cold stimulation, BA was administrated at the same time. Moreover, we found that BA can inhibit the TLR2/MYD88/NF-*κ*Bp65 signaling pathway, prevent lung inflammation, and improve lung function, to exhibit a protective effect against COPD in model rats. These results demonstrated that BA may be a potential novel drug for the treatment of COPD.

## Figures and Tables

**Figure 1:** BA improved the levels of FRC, FVC, FEV, PEF, PIF, and FEV100/FVC in the lung tissue of rats. Data were expressed as mean ± SD, *n* = 6. Compared with the control group, ^▲^*P* < 0.05 and ^▲▲^*P* < 0.01; compared with the COPD group, ^★^*P* < 0.05 and ^★★^*P* < 0.01.

**Figure 2:** BA improved the levels of TNF-*α*, IL-1*β*, IL-6, IL-8, and IL-10 in the serum of COPD rats. Data were expressed as mean ± SD, *n* = 6. Compared with the control group, ^▲^*P* < 0.05 and ^▲▲^*P* < 0.01; compared with the COPD group, ^★^*P* < 0.05 and ^★★^*P* < 0.01.

**Figure 3:** BA increased serum GSH and SOD levels and decreased MDA levels in COPD rats. Data were expressed as mean ± SD, *n* = 6. Compared with the control group, ^▲^*P* < 0.05 and ^▲▲^*P* < 0.01; compared with the COPD group, ^★^*P* < 0.05 and ^★★^*P* < 0.01.

**Figure 4:** BA improved lung histopathological changes (HE staining × 200) and semiquantitative scores in the lung tissues of COPD rats. Data were expressed as mean ± SD, *n* = 3. Compared with the control group, ^▲^*P* < 0.05 and ^▲▲^*P* < 0.01; compared with the COPD group, ^★^*P* < 0.05 and ^★★^*P* < 0.01.

**Figure 5:** BA improved the levels of TLR2, MYD88, TNF-*α*, and IL-1*β* mRNA in BALF cells of COPD rats. Data were expressed as mean ± SD, *n* = 3. Compared with the control group, ^▲^*P* < 0.05 and ^▲▲^*P* < 0.01; compared with the COPD group, ^★^*P* < 0.05 and ^★★^*P* < 0.01.

**Figure 6:** BA changed the levels of NF-*κ*B, TLR2, and MYD88 in the lung tissue of COPD rats by immunohistochemical staining and semiquantitative analysis (×100). Data were expressed as mean ± SD, *n* = 3. Compared with the control group, ^▲^*P* < 0.05 and ^▲▲^*P* < 0.01; compared with the COPD group, ^★^*P* < 0.05 and ^★★^*P* < 0.01.

**Figure 7:** BA improved the expressions of MYD88, p–NF–*κ*Bp65/NF-*κ*Bp65, p-I*κ*Ba/I*κ*Ba, TLR2, and TLR4 in rat lung tissue. Data were expressed as mean ± SD, *n* = 3. Compared with the control group, ^▲^*P* < 0.05 and ^▲▲^*P* < 0.01; compared with the COPD group, ^★^*P* < 0.05 and ^★★^*P* < 0.01.

**Table 1:** Primer sequence.

Gene	Forward primer	Reverse primer
Rat TLR2	CCCTGCTCTTTCTCACAGCA	TGACGGCCTGTATCCCTGTA
Rat MYD88	TTGGAGCCGGATTCTCCAAC	AACTGAGATGTGTGCCCAGG
Rat TNF-*α*	TGGGCTTTCGGAACTCACTG	CTGTGCCTCAGGGAACAGTC
Rat IL-1*β*	CCTTGTCGAGAATGGGCAGT	CAGGGAGGGAAACACACGTT
Rat GAPDH	TGTGAACGGATTTGGCCGTA	GATGGTGATGGGTTTCCCGT

## Data Availability

The data used to support the findings of this study are available from the corresponding author upon request.
